# A Retrospective Analysis of Internet-Based Sharing Nursing Service Appointment Data

**DOI:** 10.1155/2022/8735099

**Published:** 2022-08-18

**Authors:** Yuchen Fan, Yuezhen Ma, Yong Zhang, Changjian Sun

**Affiliations:** ^1^Department of Hepatobiliary Surgery, Shandong Provincial Third Hospital, Jinan 250000, China; ^2^Intensive Care Unit, Shandong Provincial Third Hospital, Jinan 250000, China; ^3^College of Electronic Science and Engineering, Jilin University, Changchun 130012, China

## Abstract

**Aims:**

To investigate the historical data of the “Internet+ Nursing” service platform and provide a theoretical basis to optimize the “Internet+ Nursing” service model by analyzing a population in need of nursing care services, service prices, services in demand, willingness to place orders, and feedback on use.

**Methods:**

A retrospective analysis of data related to home care services on the “Jiuzhou Nursing Care” platform from April 2020 to August 2021, a total of 279 person-times, relevant information about the research subjects, and the status of home care services was conducted. SPSS 24.0 software was used for data analyses, such as calculating frequencies and percentages and conducting chi-square tests.

**Results:**

The “Jiuzhou Online Nurse” primarily serves elderly patients, and the majority of these patients have lost their ability to care for themselves. The average cost of nursing services was ¥183.45, and the unit cost of services had no effect on the number of service items. This particular internet-based home nursing service has a high level of satisfaction. Patients aged 60 to 74 have the highest number of Internet-based home care service orders (*χ*^2^ = 11.791, *P* < 0.05). Patients who reuse the platform are more willing to assign people to provide services (*χ*^2^ = 238.078, *P* < 0.05). Patients who were unable to care for themselves had a higher rate of repeat order (*χ*^2^ = 10.877, *P* < 0.05).

**Conclusion:**

The “Internet+ Nursing” service platform specifically meets the individual needs of elderly patients, provides them with home nursing services, and improves local medical treatment and door-to-door services. This platform also provides convenience for elderly individuals who cannot care for themselves so that they can receive prompt treatment and assistance to improve their quality of life.

## 1. Introduction

As the world population continues to age, rapidly growing numbers of elderly people are exposed to risk factors for a long period of time. Due to the deterioration of organs in elderly people, physical decline, and other factors, the prevalence of chronic disease has increased. The care of discharged patients and elderly people with chronic diseases in the community have gradually become a problem that cannot be ignored [1], and growing numbers of family members have become informal caregivers, bearing large burdens of care and considerable pressure [2–4]. In this context, home care has shown positive effects, and the use of home-based long-term care services is beneficial to the health of patients with chronic diseases, especially elderly patients [5]. Home care resources may provide a more flexible and proactive approach to maintain functional status, maximize symptom relief, and prevent avoidable hospitalizations [6, 7]. Additionally, it may reduce care burden, family pressure [4, 8, 9], and medical expenditure [10]. Furthermore, home care can provide short-term care services as well as long-term healthcare services such as health exercises [11]. Professional and medically qualified family nurses can establish a harmonious relationship with the family while providing service. While providing home care services, services can be customized according to the unique needs of the family to support the effects of home care services [12–14].

In recent years, electronic and information technology have developed quickly, and a new form of “Internet +” has emerged. Medical services, including home care services, have gradually become electronic, digital, and platform-based, which has supported the integration of online and offline medical services. In developed countries, electronic and information technology are commonly used in home care. To reduce the costs of service and labor experienced as part of in-home rehabilitation, South Korea has studied the use of network-based vision and wearable device home rehabilitation systems to improve the quality of home care [15]. The United States developed internet-based care enhancement tools in the early years to build a communication bridge between consumers and medical providers [16]. Sweden uses applications as useful information and communication technology innovations that can improve communication and accessibility for older people that need home-based healthcare [17]. The Norwegian internet-based personalized online care communication platform has been successfully exposed to research on lifestyle, behavior changes, and childbirth [18–20]. Initially, China provided health guidance and online Q&A for patients with chronic diseases discharged from the hospital through mobile medical follow-up calls and official WeChat accounts [21]. In 2019, the National Health Commission announced that it would launch a pilot project with nurses [22]. As part of the “Internet +” plan, China launched the “Internet+ Nursing” service and actualized an online nursing service platform (or “online nurse appointment” platform) that allowed registered nurses to visit patients to provide home care services [23]. The online nursing service platform first started in Jinan in 2016. It has successfully expanded from Shandong Province to first-tier cities such as Beijing, Shanghai, Guangzhou, and Shenzhen [24]. The popularity of Internet in foreign countries is earlier, and the development of “Internet + nursing” platform is also earlier. For example, an Internet care platform for children with attention deficit and hyperactivity disorder (ADHD) was planned abroad in 2002 [25]. There is a platform system for a particular disease, and the platform will make personal risk reports and personal care recommendations based on the patient's daily state [26]. Although we are late in developing Internet nursing services, our platform system realizes electronization, digitization, and platformization, supporting the integration of online and offline medical services. Experience feedback is the great advantage of “Internet+ nursing” service platform. Experiential feedback helps the platform identify service deficiencies and improve the quality of home care services for patients in the community who need continuous care.

All telenurses in China are professional nursing technicians approved by medical institutions (hospitals, community healthcare centers, and private clinics). Telenurses complete personal information registration by logging into the nursing terminal of the platform. Patients can complete information registration through the client portal, apply for nursing care service, and after a shared nurse grabs (or claims) the order, the reservation is confirmed. Patients can also invite specific nurses to provide services, and the appointment is confirmed after the invitees agree. Subsequently, the shared nurse arrived at the designated place on time with the required nursing materials to complete the nursing service. After the service, the patient provides feedback regarding the nursing service.

Exploration of the patient group, service need, experience, and feedback of home care service are key roles in the “Internet+ Nursing” service for elderly patients. This research can encourage sharing of accurate information among patient groups and improve the quality of home care services for patients discharged from hospitals and patients who need continuous care in the community. On the other hand, traditional nursing care services consume considerable manpower and financial resources [27, 28]. Telenurses can meet patients' home care needs while reducing the pressure on nursing staff and appropriately allocating human resources. It determines the direction of nurses' future professional development and skill training. However, there are still few studies on patients' demand for telenurses (that is, group composition, service needs, willingness to place orders, and satisfaction). The current study is aimed at addressing the practice gap, providing a basis for improving the quality of home care, and further optimizing the shared governance model.

## 2. Materials and Methods

### 2.1. Design and Participants

The research subjects were selected patients from April 2020 to August 2021 who were discharged from hospitals, medical consortium units, and communities in Jinan City who used the “Jiuzhou Nursing Care” platform to place orders. The total number of order samples collected is 279 person-times. The inclusion criteria were as follows: register the patient's real-name information and provide a diagnosis certificate from a second-level or higher medical institution assessed by the health department.

### 2.2. Measurements

Sociodemographic information included sex, age, and self-care ability. The current status of home care services includes the itemized list of home care services, total charges, service times, order mode, order frequency, and satisfaction. The survey data come from the “Jiuzhou Nursing Care” management platform and are uniformly coded. SPSS 24.0 statistical software was used to establish a database for descriptive analysis. Statistical methods included frequency, percentage, and chi-square test. *P* < 0.05 indicates that the difference is statistically significant.

### 2.3. Quality Control

The researcher contacted the person in charge of the Jinan City “Jiuzhou Nursing Care” platform, obtained agreement, and exported relevant data content through the system. In cases of missing data, the system will prompt feedback and supplement the data in a timely manner.

## 3. Results

### 3.1. Demographic Characteristics of the Participants

The age of the study subjects was between 49 and 95 years old, with an average age of 70.96 years old. Among them, 92.8% were aged ≥60 years old, 62.0% were aged 60 to <75 years old, 29.0% were aged 75 to <90 years old, and 1.8% were aged ≥90 years old. A total of 60.6% of patients were male, and 39.4% of patients were female, as shown in Table 1.

### 3.2. “Internet+ Nursing” Home Care Service Status

The total cost of home care services in this study was ¥51183, and the number of different services for all patients was 279 person-times. The average price of the service is ¥183.45. The home care services with high demand are catheterization care, gastric tube care, and peripherally inserted central catheter (PICC) maintenance. Oral care and tracheotomy care services were the least common. The project with the highest average price is pressure ulcer wound care, and the price is ¥258. The lowest average price item is venous blood collection, and the price is ¥162.  Table 2 shows the payment status of home care service orders for research subjects.

The satisfaction with home care services was as high as 100%, and 98.6% of patients who received home care services were very satisfied, as shown in Table 3.

Differences in order mode selection among patients of different ages include the following: patients between the ages of 60 and 74 have the largest number of home care orders and patients over 90 years old have the least number of home care orders. The home care service order mode in this study is divided into two modes: grab order mode and designated mode. Most of the order modes were grabbing orders. For patients aged 60 to 89, the proportion of designated orders increases gradually with the increase of age. There was a significant correlation between age and order mode (*P* < 0.05), as shown in Table 4.

The home care service order frequency in this study includes multiple orders and a single order. As shown in Table 5, the same registered user places 37.99% of orders multiple times. Differences in order mode selection among patients with different order frequencies include a total of 97.7% of patients who ordered only one home care service with the same registered account chose the order-grabbing mode, while 94.3% of patients who ordered home care services with the same registered account multiple times chose the designated service provider for nursing care. Patients who only seek home care are more inclined to designate personnel to provide onsite services.

There was a significant correlation between order frequency and order mode (*P* < 0.05), as shown in Table 6. The Pearson between order frequency and order mode is 0.385, and the *P* value is less than 0.05, the positive correlation between order frequency and order mode is significant. This indicates that users with more orders tend to prefer the specified order mode.

As shown in Table 7, patients with total loss of self-care ability placed orders the most frequently, accounting for 65.9% of the total number of orders. Patients with partial loss of self-care ability accounted for 26.2% of the total, and patients with self-care ability placed the least orders. Additionally, patients with total loss of self-care ability had the highest proportion of multiple orders, accounting for 75.5%.

There was no significant correlation between order frequency and self-care ability (*P* > 0.05), as shown in Table 8. The Pearson between order frequency and self-care ability is only -0.061; *P* value is greater than 0.05, so the correlation between order frequency and self-care ability is not significant.

## 4. Discussion

The composition of family nursing service demand groups is the research object of this study. The analysis and discovery of service groups will optimize the nursing service mode in the next step. In order to better study the difference of the elderly, the age was grouped according to the new age segmentation of the World Health Organization [29]. As shown in Table 1, the average age of patients with chronic diseases in this survey was 70.96 years old, of which 92.8% were aged ≥60 years old, indicating that elderly patients with chronic diseases are the main group demanding home care services, and they are not excluded from accepting internet appointments for home care services because they are not familiar with the internet. Although some elderly patients are unable to operate their mobile phones proficiently [30, 31], they still have the opportunity to reserve care services via the internet with the help of their family members.

Analyzing the popularity of different services from the perspective of home care services can provide data support for medical institutions in the cultivation of professional talent and the deployment of medical resources. As shown in Table 2, the services with high demand in this study are catheterization care, gastric tube care, and PICC catheter maintenance, followed by pressure ulcer wound care, sputum suction care, and venous blood sampling, which indicates that the most frequently requested home care services are medical services. On the one hand, high-demand services require highly skilled professionals, and while nursing materials are difficult to obtain, families experience difficulty in providing care independently. Therefore, support from professional and technical personnel is required. Second, high-demand services are common for diseases that require long-term treatment and recovery, which increases the frequency of patients' needs. Especially in the context of shortened hospital stays and improved community health services, communities and family homes have become the main places for the treatment and rehabilitation of most chronic diseases, and the demand for professional nursing care services is increasing among elderly patients. This has increased the urgency of seamless connection between home care and hospital care. Providing professional and appropriate treatment and nursing care technology is the basis for satisfactory home care services for elderly patients with chronic diseases [32].

Economic pressure is a factor that affects home care services. Patients with chronic disease have a long course of illness and a high treatment costs, which increases the financial burden on the family and affects the patient's ability and willingness to pay their bills. This study analyzes the relationship between the average price of a single service and the number of services to identify whether the patient group has a low willingness to pay for home care, which restricts the development of home care services. As shown in Table 2, the average price of the services in this study is RMB 183.45. At present, home care services are not included in medical insurance and but are instead paid at the patients' expense. It is worth noting that after comparing and analyzing the service times and prices of different projects, we found that the times of different services did not have a positive correlation with service prices. This may depend on two reasons: first, because home care does not need to occupy the space of a medical institution and can flexibly occupy other locations, the price is much lower than the cost of nursing care in a medical institution [33]; second, because most medical services are necessary expenses for families, the development of home care services is not restricted. However, improving the “Internet+ Nursing” service platform, reducing service costs to provide professional and appropriate nursing care services, reducing the burden of care for family members, and meeting home care service needs for elderly patients with chronic diseases are still important goals for this service model.

The service satisfaction data reveal that patients are highly satisfied with online appointment care. As shown in Table 3, 98.6% of patients reported that they were very satisfied with the service. High levels of satisfaction encourage patients to make repeat appointments on the platform. As shown in Tables 3 and 4, when analyzing order frequencies, repeat orders accounted for 37.99%, and the number of elderly patients with chronic diseases between age 60 and 74 who placed home care orders was the largest. This shows that “young elderly” individuals [34] have a higher demand for home care services, which indicates that young elderly individuals are better at accepting and applying via medical websites, apps, hospital WeChat public accounts, and other service platforms to obtain relevant medical service information. From the order mode perspective, there is a significant correlation between age and order mode. As shown in Tables 4 and 5, the older people are, the higher the proportion of making orders. As they grow older, they become more isolated and require customized nursing care services. Appointing people who are more familiar with their condition to make an appointment for nursing care services will be more beneficial to their care. In addition, people who repeatedly place orders are more likely to choose a dedicated service provider, indicating their demand for and affirmation of the professional skills of nursing staff.

The home care appointment model is of great significance to patients who lack total self-care ability. As shown in Table 7, patients with chronic diseases who have lost their ability to care for themselves place the most frequent orders, and the proportion of multiple orders is the highest [35]. The proportion of people who could not care for themselves was 92.1%. As age increases, physical functions decline, and the demand for home care services increases. Elderly people who cannot care for themselves need targeted care services [36]. This shows that the home care service model has significantly improved the convenience of nursing care for this group. This portion of the population does not require hospital care; they can easily receive home care instead.

## 5. Limitations

This study has limitations. First, the research subjects included in this study were all from hospitals, medical union units, and communities in Jinan, which limits the generalizability of the results. Second, this study only performed a descriptive analysis of the current status of the use of services for people who have ordered home care services and did not identify the factors that influence home care services and the nurses using the platform. These two limitations can be addressed in future studies to provide sufficient evidence to improve practice.

## 6. Conclusion

The “Internet+ Nursing” service based on the online nurse appointment platform is a new intelligent nursing care model. Through a retrospective analysis of the order data of “Jiuzhou Nursing”, including the patient's gender, age, self-care ability, home care service items, cost, order method, order time, and satisfaction, this study found that the platform can provide personalized services to patients' needs. Through resource integration, information sharing, and convenient use, this platform provides seamless connection between home care and hospital care. Elderly patients are the main group demanding home care service, especially elderly patients who are unable to care for themselves. The demand is mainly for professional nursing care, and the price of service is lower than the price of hospital care. Feedback regarding services indicate a high level of satisfaction, and patients are more willing to allow the people they are familiar with to provide care services. On the other hand, through the “Internet+ nursing” service, the pressure on nursing staff can be reduced, and human resources can be appropriately allocated. Research on the current status of services from the patients' perspective provides theoretical guidance to optimize service models.

## Figures and Tables

**Table 1:** Relevant situation of research subjects (*n* = 279).

		Count (*n*)	Percent (%)
Gender	Male	169	60.6%
	Female	110	39.4%

Age group (years)	<60	20	7.2%
	60 to <75	173	62.0%
	75 to <90	81	29.0%
	≥90	5	1.8%

**Table 2:** Payment status of home care service orders for research subjects (*n* = 279).

Service items	Service charge (¥)	Service times (*n*)	Average price (¥)
PICC maintenance	7378	31	238
Bladder irrigation	334	2	167
Catheterization care	18512	104	178
Enema care	609	3	203
Venous blood collection	810	5	162
Oral care	178	1	178
Tracheostomy care	218	1	218
Surgical wound dressing	344	2	172
Stomach tube care	19040	112	170
Sputum suction care	1008	6	168
Pressure ulcer wound care	2064	8	258
Stoma care	688	4	172

**Table 3:** Research subjects' home care service orders and satisfaction (*n* = 279).

Satisfaction degree	Count (*n*)	Percent (%)
Very dissatisfied	0	0.0%
Dissatisfied	0	0.0%
Generally	0	0.0%
Satisfy	4	1.4%
Very satisfied	275	98.6%

**Table 4:** Comparison of ordering modes among patients of different age groups (*n* = 279).

Group	Order mode				Chi-square	*P* value
	Grab an order, *N* (%)		Specify, *N* (%)			
Age (years)					11.791	0.006
<60	19	95.0%	1	5.0%		
60 to <75	107	61.8%	66	38.2%		
75 to <90	46	56.8%	35	43.2%		
≥90	3	60.0%	2	40.0%		
Total	175	62.7%	104	37.3%		

**Table 5:** Comparison of patient ordering modes with different ordering frequencies (*n* = 279).

Group	Order mode				Total		Chi-square	*P* value
	Grab an order, *N* (%)		Specify, *N* (%)					
Frequency							238.078	0.001
Single	169	97.7%	4	2.3%	173	62.01%		
Multiple	6	5.7%	100	94.3%	106	37.99%		
Total	175	62.7%	104	37.3%	279	100%		

**Table 6:** Correlation analysis between order frequency and order mode (*n* = 279).

		Order mode
Order frequency	Pearson	0.385^∗∗^
	Significant difference	0.000
	Total	279

^∗∗∗^ *P* < 0.01, ^∗∗^*P* < 0.05, and ^∗^*P* < 0.1.

**Table 7:** Comparison of ordering frequencies of patients with different self-care abilities (*n* = 279).

Group	Self-care ability						Chi-square	*P* value
	Self-care, *N* (%)		Partial loss, *N* (%)		Complete loss, *N* (%)			
Frequency							10.877	0.004
Single	12	6.9%	57	32.9%	104	60.1%	173	
Multiple	10	9.4%	16	15.1%	80	75.5%	106	
Total	22	7.9%	73	26.2%	184	65.9%	279	

**Table 8:** Correlation analysis between order frequency and self-care ability (*n* = 279).

		Self-care ability
Order frequency	Pearson	-0.061
	Significant difference	0.307
	Total	279

## Data Availability

The data used to support the findings of this study are included in the article.

## Supplementary Materials

Supplementary Materials The ethical approval document and English translation version.
